The article "Clinicopathological and Prognostic Significance of PRAME Overexpression in Human Cancer: A Meta-Analysis" was published in 2020. Journal: Biomed Res Int.

# Clinicopathological and Prognostic Significance of PRAME Overexpression in Human Cancer: A Meta-Analysis

**DOI:** 10.1155/2020/8828579

**Published:** 2020-12-11

**Authors:** Jiaqiang Li, Jianchun Yin, Jianhua Zhong, Zhilin Yang, Aifa Tang, Shoulin Li

**Affiliations:** ^1^Department of Pediatric Urology, Shenzhen Children's Hospital, Shenzhen, Guangdong 518026, China; ^2^Department of Science and Education, The Second People's Hospital of Shenzhen, The First Affiliated Hospital of Shenzhen University, Shenzhen, Guangdong 518035, China

## Abstract

Numerous studies have demonstrated that preferentially expressed antigen in melanoma (PRAME) is abnormally expressed in various solid tumours. However, the clinicopathological features and prognostic value of the PRAME expression in patients with cancer remain unclear. Accordingly, we performed a meta-analysis to accurately assess the association of the expression level of PRAME with clinicopathological features and cancer prognosis. Relevant study collection was performed in PubMed, Web of Science, and Embase until 28 February 2020. A total of 14 original studies involving 2,421 patients were included. Our data indicated that the PRAME expression was significantly associated with tumour stage (OR = 1.99, 95% CI: 1.48–2.67, *P* < 0.001) and positive lymph node metastasis (OR = 3.14, 95% CI: 1.99–4.97, *P* < 0.001). Pooled results showed that overexpression of PRAME is positively correlated with poor disease-free survival (HR = 1.60, 95% CI: 1.36–1.88, *P* < 0.001), progression-free survival (HR = 1.88, 95% CI: 1.02–3.46, *P* = 0.042), metastasis-free survival (HR = 1.86, 95% CI: 1.05–3.31, *P* = 0.034), and overall survival (HR = 1.75, 95% CI: 1.53–1.99, *P* < 0.001). In summary, these data are suggesting that PRAME is tumorigenic and may serve as a prognostic biomarker for cancer.

## 1. Background

Cancer has become a major public health problem worldwide. According to a previous study, approximately 1,735,350 new cancer cases and 609,640 million cancer deaths occurred in the United States in 2018 [1]. Despite medical and scientific efforts over the past decades, the overall 5-year survival rate remains low because of the malignant progression of tumours [1]. Biomarkers have become important tools for tumour diagnosis, and they also serve as therapeutic targets and can be used to predict clinical outcomes [2]. Therefore, identifying potential novel biomarkers is imperative for refining and optimizing diagnosis, treatment, and prognosis.

Cancer/testis antigens (CTAs) represent a heterogeneous group of tumour antigens and are regarded as ideal potential biomarkers for detection and targets in cancer immunotherapy because of their restricted expression pattern and immunogenicity [3]. In recent years, several CTAs have been studied as target antigens in vaccine clinical trials for various cancer types [4]. Preferentially expressed antigen in melanoma (PRAME) is one of the most immunogenic CTAs discovered to date. The PRAME protein was first described as a tumour antigen in human melanoma by Ikeda et al. [5]. Subsequently, numerous studies reported that overexpression of PRAME was significantly correlated with clinicopathological features in malignant tumours, including medulloblastoma [6], hepatocellular carcinoma [7, 8], adenocarcinoma [9], uveal melanoma [10, 11], high-grade serous cancer [12], myxoid liposarcoma [13], diffuse large B-cell lymphoma [14], osteosarcoma [15], bladder cancer [16], breast carcinoma [17, 18], and neuroblastoma [19]. However, the consistency of the clinicopathological features and prognostic value of PRAME remains unclear.

To our knowledge, this meta-analysis is the first complete overview to clarify the clinicopathological features and prognostic value of PRAME based on the information from all previously published studies.

## 2. Materials and Methods

### 2.1. Search Strategy

In accordance with the PRISMA statement, we conducted a systematic literature search of PubMed, Web of Science, and Embase using “PRAME” OR “preferentially expressed antigen in melanoma” as keywords. The search concluded in this study was updated in February 2020. We manually reviewed the references of the retrieved articles to identify potentially eligible studies.

### 2.2. Selection Criteria

Eligible articles met the inclusion criteria based on the following: (1) articles assessed the prognostic or clinical value of PRAME in solid tumours, (2) articles published in English, and (3) articles provided odds ratios (ORs) or information that allowed manual calculation of the 95% confidence intervals (CIs). The articles excluded were (1) duplicated publications; (2) reviews, comments, letters, and conference abstract; (3) and articles without usable data.

### 2.3. Data Extraction

Two investigators extracted the data from selected studies independently, including the first author's name, year of publication, country, cancer type, number of cases, detection method, tumour stage, number of patients with positive PRAME and negative PRAME expression, HRs, and 95% CIs for DFS, PFS, MFS, and OS. The HRs and 95% CIs were directly extracted from the adequate information in the article; otherwise, we used the Engauge Digitizer version 4.1 software to estimate the survival data from Kaplan-Meier curves.

### 2.4. Statistical Analysis

The quality of the selected studies was independently evaluated by two reviewers using the Newcastle-Ottawa Scale (NOS). All statistical analyses were performed using the Stata statistical software version 14.0 (Stata Corporation, College Station, TX, USA). Heterogeneity among studies was assessed using Cochrane's *Q* tests (chi-squared tests) and the *I*^2^ statistic. The fixed-effects model was adopted when there was no obvious heterogeneity (*P* > 0.1 and *I*^2^ < 50%). Otherwise, a random-effects model was applied. Egger's test was used to assess publication bias. Sensitivity analysis was conducted to investigate the stability of the total pooled results by removing studies one by one. *P* < 0.05 was considered statistically significant.

## 3. Results

### 3.1. Study Selection and Characteristics

The flow diagram is shown in Figure 1; a total of 1,149 articles were identified for initial evaluation, and 1,087 manuscripts were excluded from analysis because of irrelevant titles or duplicates. We excluded 32 citations based on their abstracts, leaving 30 studies for further full-text review. After further reading of the studies, we excluded 16 studies because of insufficient survival data. Ultimately, 14 studies meeting the selection criteria were finally included in this meta-analysis.

The main features of the 14 eligible studies are summarized in Table 1. The publication years of the eligible studies ranged from 2004 to 2019. The total number of patients was 2,421 with a mean of 172.9 (range, 51–576 patients). Among the 14 studies, one focused on medulloblastoma, two on hepatocellular carcinoma, one on adenocarcinoma, two on uveal melanoma, one on high-grade serous cancer, one on myxoid liposarcoma, one on diffuse large B-cell lymphoma, one on osteosarcoma, one on bladder cancer, two on breast carcinoma, and one on neuroblastoma. Eleven of the studies evaluated PRAME at the gene level, while four conducted evaluation at the protein level. Patients were dichotomized into two groups with positive and negative PRAME expression. The quality of the selected studies was assessed by using the Newcastle-Ottawa Scale and found to range from 6 to 8, indicating that the studies were of good quality.

### 3.2. Meta-Analysis Results

#### 3.2.1. PRAME Expression and Clinicopathological Parameters

Nine articles investigated the associations between PRAME expression and tumour stage. There were 604 cases of III–IV stage and 559 cancer cases of I–II stage (Table 1). Since the low heterogeneity (*I*^2^ = 43.4%, *P* = 0.079), we used the fixed-effects model to pool data. The stratified data showed that the PRAME overexpression was significantly associated with tumour stage (OR = 1.99, 95% CI: 1.48–2.67, *P* < 0.001) (Figure 2(a)). The results suggest that the increased expression of PRAME was markedly higher in the III–IV stage group than in the I–II stage group.

Four articles investigated the associations between PRAME expression and lymphatic metastasis. These were 158 cases of positive lymphatic metastasis and 190 cases of negative lymphatic metastasis (Table 1). Since the low heterogeneity (*I*^2^ = 8.8%, *P* = 0.349), we used the fixed-effects model to pool data. The stratified data showed that the PRAME overexpression was significantly associated with lymphatic metastasis (OR = 3.14, 95% CI: 1.99–4.97, *P* < 0.001) (Figure 2(b)). The results indicate that the increased expression of PRAME was markedly higher in the positive lymphatic metastasis group than in the negative lymphatic metastasis group.

#### 3.2.2. Correlation between the PRAME Expression and Disease-Free Survival (DFS)

There were four studies, comprising a total of 858 patients, provided data for us to analyse the correlation between PRAME and DFS. Since the low heterogeneity (*I*^2^ = 28.9%, *P* = 0.239), we used the fixed-effects model to pool data. As seen in Figure 3(a), the data indicated that the overexpression of PRAME had an obvious impact on DFS (HR = 1.60, 95% CI: 1.36–1.88, *P* < 0.001). The overall results suggest that PRAME overexpression is an indicator of poor DFS in patients with cancer.

#### 3.2.3. Correlation between the PRAME Expression and Progression-Free Survival (PFS)

There were three studies, comprising a total of 603 patients, provided data for us to analyse the correlation between PRAME and PFS. Since the low heterogeneity (*I*^2^ = 0.0%, *P* = 0.375), we used the fixed-effects model to pool data. As seen in Figure 3(b), the data indicated that the overexpression of PRAME had an obvious impact on PFS (HR = 1.88, 95% CI: 1.02–3.46, *P* = 0.042). The overall results suggest that PRAME overexpression is an indicator of poor PFS in patients with cancer.

#### 3.2.4. Correlation between the PRAME Expression and Metastasis-Free Survival (MFS)

There were four studies, comprising a total of 689 patients, provided data for us to analyse the correlation between PRAME and MFS. Since the obvious heterogeneity (*I*^2^ = 89.7%, *P* ≤ 0.001), we used the random-effects model to pool data. As seen in Figure 3(c), the data indicated that the overexpression of PRAME had an obvious impact on MFS (HR = 1.86, 95% CI: 1.05–3.31, *P* = 0.034). The overall results suggest that PRAME overexpression is an indicator of poor MFS in patients with cancer.

#### 3.2.5. Correlation between the PRAME Expression and Overall Survival (OS)

There were twelve studies, comprising a total of 1,978 patients, provided data for us to analyse the correlation between PRAME and OS. Since the low heterogeneity (*I*^2^ = 46.5%, *P* = 0.038), we used the fixed-effects model to pool data. As seen in Figure 3(d), the data indicated that the overexpression of PRAME had an obvious impact on OS (HR = 1.75, 95% CI: 1.53–1.99, *P* < 0.001). The overall results suggest that PRAME overexpression is an indicator of poor OS in patients with cancer.

Because of heterogeneity in the samples, subgroup analysis was performed for study location, sample size, and testing index (Table 2). There was an obvious relationship between the high expression of PRAME and shorter OS in Asian patients with cancer (HR = 1.41, 95% CI: 1.02–1.95, *P* < 0.001) and non-Asian patients with cancers (HR = 2.36, 95% CI: 1.81–3.08, *P* < 0.001). Meanwhile, there was an obvious relationship between the high PRAME expression and the OS of patients with sample sizes of ≥100 (HR = 1.49, 95% CI: 1.04–2.15, *P* < 0.001) and <100 (HR = 2.14, 95% CI: 1.60–2.85, *P* < 0.001). In addition, there was an obvious relationship between the high PRAME expression and the OS of patients with different testing methods (qRT-PCR: HR = 1.691, 95% CI: 1.016–2.814, *P* = 0.043; IHC: HR = 1.784, 95% CI: 1.186–2.685, *P* = 0.005; microarray: HR = 1.752, 95% CI: 1.186–2.685, *P* < 0.001).

### 3.3. Publication Bias

Publication bias was evaluated by funnel plot and Egger's test. Because of the small sample size of LNM, DFS, PFS, and MFS, we had not conducted publication bias analysis. The results indicated no significant publication bias was observed in this analysis (Figure 4).

### 3.4. Sensitivity Analysis

Sensitivity analysis was performed to assess the influence of each study omission on the overall outcome. The results suggested that there was no significant influence of the pooled HR by omitting any study, indicating our analysis was robust (Figure 5).

## 4. Discussion

There is growing evidence that the overexpression of PRAME can contribute to the differences in the prognostic outcome between different kinds of solid tumors. To the best of our knowledge, this study describes the first meta-analysis to analyse the association between the level of PRAME and the clinicopathological features and prognostic value of patients in solid tumours comprehensively and systematically. In this study, we included 14 retrospective studies with a total of 2,421 patients. Remarkable positive associations were identified between the PRAME expression and clinicopathological characteristics, including advanced clinical stage (*P* < 0.001) and positive lymph node metastasis (*P* < 0.001). The results of the overall analysis revealed that the overexpression of PRAME is positively related to poor DFS (*P* < 0.001), PFS (*P* = 0.042), MFS (*P* = 0.034), and OS (*P* < 0.001). The results of the heterogeneity in the subgroup analyses also showed that our results were stable for all variables. Therefore, these results indicated that PRAME might serve as a clinicopathological and prognostic biomarker for malignancy.

Numerous studies have reported PRAME expression in various malignancies. In solid malignancies, including hepatocellular carcinoma [7, 8], uveal melanoma [10, 11], osteosarcoma [15], bladder cancer [16], and breast carcinoma [18], high PRAME expression correlates with advanced-stage disease and poor survival, whereas in pediatric acute leukemia, PRAME overexpression was found to predict good outcome [20–22]. Steinbach et al. [21] found that the overexpression of PRAME was found in 62% (*n* = 31) of acute myeloid leukemia patients, and the rates of OS and DFS were higher than in patients with no or low expression (*P* < 0.05). Moreover, Abdelmalak et al. [20] reported that positive PRAME expressers had a statistically longer DFS and OS (*P* < 0.001, <0.001, respectively) compared with negative PRAME expressers. These studies suggest that PRAME overexpression is a predictor for better prognostic outcome in acute leukemia, which is completely opposite to the prognostic results of solid tumors in our meta-analysis. However, large-scale and prospective cohort studies will ultimately be needed to validate the good prognostic outcome of PRAME overexpression in acute leukemia.

As we all know, DNA methylation is an epigenetic mechanism often affecting gene expression and modifying the function of the genes. PRAME has been reported to be epigenetically regulated by DNA methylation in malignancies. Field et al. [11] found that PRAME is aberrantly hypomethylated and transcriptionally activated in uveal melanomas and is associated with increased metastatic risk. Moreover, PRAME is frequently expressed in epithelial ovarian cancer at the mRNA and protein levels, and DNA methylation is a key mechanism regulating its expression [12]. Additionally, Schenk et al. [23] reported that changes in the methylation pattern in defined parts of the regulatory regions of PRAME are sufficient for its upregulation in cells. Together, these studies show that the PRAME expression is associated with aberrant hypomethylation of the PRAME promoter and may have therapeutic implications. To note, most of the studies included in this meta-analysis have not identified the association between PRAME promoter DNA hypomethylation and its expression, which warrants further investigations.

Although the function of PRAME has not yet been fully elucidated, a number of studies have addressed this issue. It is known that PRAME can bind to the retinoic acid receptor in the presence of retinoic acid, which suggests that it serves as a transcription regulator of nuclear receptor signaling [24]. PRAME knockdown was shown to decrease the proliferation of cancer cells [7, 15, 24, 25]. Tan et al. [15] found that PRAME siRNA knockdown significantly suppressed the proliferation, colony formation, and G1 cell cycle arrest in primary osteosarcoma. Oehler et al. [25] reported that PRAME inhibits myeloid tumor cell differentiation in leukemic progenitor cells. Downregulation of PRAME suppresses proliferation and promotes apoptosis in hepatocellular carcinoma through the activation of the P53-mediated pathway [7]. Additionally, Orlando et al. [6] reported that high PRAME mRNA expression correlates significantly with a worse OS and PRAME-specific TCR may represent a promising innovative approach for treating medulloblastoma patients. To date, PRAME is one of the most immunogenic CTAs discovered thus far, regarding as an attractive potential immunotherapy target [4, 26–28]. The vaccination approaches using PRAME as the target are currently undergoing clinical trials (trial numbers NCT01149343, NCT01853878, and NCT00423254) [27].

There were several limitations in this study that should be acknowledged. Firstly, the articles included were from only three databases (PubMed, Web of Science, and Embase); thus, the data collection may be incomplete. Secondly, different criteria were applied in these studies for defining PRAME positive or negative, because of the lack of uniform cut-off values in PRAME expression. Thirdly, HRs with 95% CIs were calculated by digitizing and extracting from the survival curves in several papers, which inevitably brought minor statistical deviations. Furthermore, the effects of some factors, such as age and gender, were not considered in this analysis because of insufficient data. Therefore, high-quality studies are urgently needed to draw more accurate conclusions.

Our meta-analysis provided credible evidence that the overexpression of PRAME was significantly related to the TNM stage, LNM, and poor prognosis. In addition, PRAME might serve as an attractive therapeutic target in the treatment of malignant tumors. However, considering the limitations of individual study, large-scale and prospective cohort studies will ultimately be needed to validate the results of our study.

## Figures and Tables

**Figure 1:** Flow diagram of the study selection in the meta-analysis.

**Figure 2:** Forest plot of studies evaluating the associations between the PRAME overexpression and clinicopathological features. (a) Tumor stage: III+IV. (b) Lymph node metastasis: present.

**Figure 3:** Forest plot of studies evaluating the associations between the PRAME overexpression and prognostic features. (a) DFS. (b) PFS. (c) MFS. (d) OS.

**Figure 4:** Funnel plot for publication bias in PRAME-related studies. (a) Tumor stage. (b) OS.

**Figure 5:** Sensitivity analyses of the studies. (a) Tumor stage. (b) OS.

**Table 1:** Main characteristics of 14 studies included in the meta-analysis.

Study	Year	Country	Cancer type	Number	Gene (+/-) no.	Detection method	Tumor stage	Lymphatic metastasis	Analysis method	Survival analysis	HR statistic	Hazard ratios (95% CI)	NOS scale
							I+II/III+IV	Yes/no					
Orlando et al. [6]	2018	Italy	MB	51	19/32	RT-qPCR	NR	NR	NR	OS	Rep	4.26 (2.23, 15.39)	7
Zhu et al. [7]	2018	China	HCC	96	58/38	IHC	59/37	40/56	NR	OS, MFS	Rep	1.46 (0.47, 2.93) 1.04 (1.01, 1.09)	8
Pan et al. [9]	2017	Taiwan, China	AC	156	39/82	RT-qPCR	84/37	NR	NR	OS	Rep	0.36 (0.27, 1.66)	7
Gezgin et al. [10]	2017	Netherlands	UM	64	29/35	Microarray	41/23	37/17	NR	OS	SC	1.98 (0.96, 4.08)	7
Field et al. [11]	2016	Netherlands	UM	203	51/152	RT-qPCR and RNA-Seq	NR	NR	MA	OS, MFS	SC	2.33 (1.83, 4.19) 2.51 (1.71, 7.14)	7
Oyama et al. [8]	2016	Japan	HCC	100	27/73	RT-qPCR	57/43	NR	NR	OS, DFS	SC	1.28 (0.82, 1.98) 1.42 (0.92, 2.21)	7
Zhang et al. [12]	2016	USA	HGSC	576	288/288	Microarray	NR	NR	NR	OS, DFS	SC	1.70 (1.42, 2.04) 1.54 (1.28, 1.86)	8
Iura et al.[13]	2015	Japan	MLS	79	44/35	IHC	NR	NR	MA	OS, DFS	SC	1.60 (0.44, 5.89) 1.93 (0.73, 5.07)	6
Mitsuhashi et al.[14]	2014	Japan	DLBCL	160	21/139	IHC	75/85	NR	UA	OS, PFS	Rep	1.89 (0.7, 4.34) 2.40 (1.12, 4.67)	7
Tan et al.[15]	2012	China	Osteosarcoma	95	32/63	IHC	84/10	23/72	NR	OS, MFS	Rep	1.93 (1.08, 3.43) 2.76 (1.65, 4.61)	8
Dyrskjot et al. [16]	2012	Denmark	BC	349	71/278	RT-qPCR	78/253	NR	UA	PFS	Rep	0.61 (0.08, 4.61)	7
Epping et al.[17]	2008	Netherlands	BCA	295	98/197	RT-qPCR	NR	NR	MA	OS, MFS	SC	2.31 (1.43, 3.72) 1.99 (1.33, 2.99)	8
Doolan et al.[18]	2008	Ireland	BCA	103	55/48	RT-qPCR	50/53	58/45	UA	OS, DFS	SC	2.00 (0.69, 5.75) 3.04 (1.57, 5.88)	8
Oberthuer et al.[19]	2004	Germany	Neuroblastoma	94	74/20	Northern blotting	31/63	NR	NR	PFS	SC	1.24 (0.30, 5.17)	6

MB: medulloblastoma; HCC: hepatocellular carcinoma; AC: adenocarcinoma; UM: uveal melanoma; HGSC: high-grade serous cancer; MLS: myxoid liposarcoma; DLBCL: diffuse large B-cell lymphoma; BC: bladder cancer; BCA: breast carcinoma; IHC: immunohistochemistry; RT-qPCR: quantitative real-time PCR; NR: not reported; UA: univariate analysis; MA: multivariate analysis; OS: overall survival; MFS: metastasis-free survival; DFS: disease-free survival; PFS: progression-free survival; HR: hazard ratio; Rep: reported; SC: survival curve; CI: confidence interval; NOS: Newcastle-Ottawa scores.

**Table 2:** Subgroup analysis of the studies reporting the association of overexpression of PRAME and OS of cancer patients.

Stratified analysis	No. of studies	No. of patients	Pooled HRs (95% CI)		*P* value	Heterogeneity	
			Fixed	Random		*I* ^2^ (%)	*P* value
Study location							
Asia	7	1262	1.58 (1.36, 1.84)	1.41 (1.02, 1.95)	<0.001	51.3	0.06
Non-Asia	5	716	2.36 (1.81, 3.08)	2.36 (1.81, 3.08)	<0.001	0	0.78
Sample size							
≥ 100	6	1298	1.65 (1.42, 1.92)	1.49 (1.04, 2.15)	<0.001	66.8	0.01
<100	6	680	2.14 (1.60, 2.85)	2.14 (1.60, 2.85)	<0.001	0	0.69
Index							
qRT-PCR	6	908	1.79 (1.42, 2.26)	1.69 (1.02, 2.81)	0.043	75	0.01
IHC	4	430	1.78 (1.19, 2.69)	1.78 (1.19, 2.69)	0.005	0	0.96
Microarray	2	640	1.72 (1.44, 2.05)	1.72 (1.44, 2.05)	<0.001	0	0.69

## Data Availability

All data used to support the findings of this study are included within the article.

## Abbreviations

CTAs: Cancer/testis antigens
PRAME: Preferentially expressed antigen in melanoma
MB: Medulloblastoma
HCC: Hepatocellular carcinoma
AC: Adenocarcinoma
UM: Uveal melanoma
HGSC: High-grade serous cancer
MLS: Myxoid liposarcoma
DLBCL: Diffuse large B-cell lymphoma
BC: Bladder cancer
BCA: Breast carcinoma
IHC: Immunohistochemistry
RT-qPCR: Quantitative real-time PCR
NR: Not reported
UA: Univariate analysis
MA: Multivariate analysis
OS: Overall survival
MFS: Metastasis-free survival
DFS: Disease-free survival
PFS: Progression-free survival
HR: Hazard ratio
Rep: Reported
SC: Survival curve
CI: Confidence interval
NOS: Newcastle-Ottawa scores.
